The article "Influence of Two Common Polymorphisms in the EPHX1 Gene on Warfarin Maintenance Dosage: A Meta-Analysis" was retracted in 2019. Reasons: errors in the analysis; plagiarism; overlap with other authors' work; false authorship.

# Influence of Two Common Polymorphisms in the *EPHX1* Gene on Warfarin Maintenance Dosage: A Meta-Analysis

**DOI:** 10.1155/2015/564149

**Published:** 2015-01-06

**Authors:** Hong-Qiang Liu, Chang-Po Zhang, Chang-Zhen Zhang, Xiang-Chen Liu, Zun-Jing Liu

**Affiliations:** ^1^Department of Pharmacy, Jining No. 1 People's Hospital, Jining 272011, China; ^2^Jining Hospital of Traditional Chinese Medicine, Jining 272137, China; ^3^Jining Municipal Authority Hospital, Jining, Shandong 272000, China; ^4^Department of Neurology, China-Japan Friendship Hospital, Yinghua Road No. 2, Chaoyang District, Beijing 100029, China

## Abstract

We conducted a meta-analysis to investigate the influence of two common single nucleotide polymorphisms (SNPs) (rs2292566 G>A and rs4653436 A>G) in the *EPHX1* gene on warfarin maintenance dosages. Relevant literatures were searched using the *PubMed, Embase, Web of Science, Cochrane Library, CISCOM, CINAHL, Google Scholar, CBM*, and *CNKI* databases without any language restrictions. STATA Version 12.0 software (Stata Corporation, College Station, TX, USA) was used for this meta-analysis. Standard mean difference and its corresponding 95% confidence interval (95% CI) were calculated. Seven studies met the inclusion criteria, including 2,063 warfarin-treated patients. Meta-analysis results illustrated that *EPHX1* rs2292566 G>A polymorphism might be strongly correlated with a higher maintenance dose of warfarin. However, no interaction of *EPHX1* rs4653436 A>G polymorphism with warfarin maintenance dosage was detected. A further subgroup analysis based on stratification by ethnicity indicated that *EPHX1* rs2292566 G>A polymorphism was positively correlated with warfarin maintenance dosage among Caucasians, but not Asians. No associations were observed between *EPHX1* rs4653436 A>G polymorphism warfarin maintenance dosage among both Caucasians and Asians. Our meta-analysis provides robust and unambiguous evidence that *EPHX1* rs2292566 polymorphism may affect the maintenance dose of warfarin in Caucasians.

## 1. Introduction 

Warfarin is an anticoagulant normally involved in preventing thrombosis and thromboembolism, which is prescribed for patients with chronic atrial fibrillation, pulmonary embolism, deep vein thrombosis, recurrent stroke, and prosthetic heart valves [1–4]. In clinical practice, warfarin anticoagulant activity should be monitored for the international normalized ratio (INRs) to ensure an appropriate, safe, and efficient dose; incorrect dosage administration may cause a high risk of potentially devastating bleeding and failure of preventing thrombosis [5–7]. Several factors have been reported to influence the variability in warfarin dose, including age, body size, vitamin K intake, interacting medications, and genetic variants [8–11]. A large number of evidences demonstrated that genotype-guided dosing of warfarin is a widely recognized example of pharmacogenetics, and clinical utility of genetics-guided warfarin initiation would provide safe and optimal anticoagulation therapy [12, 13].

The article "Influence of Two Common Polymorphisms in the EPHX1 Gene on Warfarin Maintenance Dosage: A Meta-Analysis" was retracted in 2019. Reasons: errors in the analysis; plagiarism; overlap with other authors' work; false authorship.

Recent studies suggested that microsomal epoxide hydrolase 1 (EPHX1) may alter the pharmacokinetics and pharmacodynamics of warfarin and have a clinically significant impact on warfarin maintenance dose [14, 15]. EPHX1 is a critical xenobiotic-metabolizing enzyme, catalyzing both detoxification and bioactivation reactions that direct the disposition of chemical epoxides including the carcinogenic metabolites of several polycyclic aromatic hydrocarbons [16, 17]. To the best of our knowledge, EPHX1 plays an important role in the majority of xenobiotic metabolisms and ensures widespread defense against potentially genotoxic epoxide intermediates including vitamin K epoxide, which is attributed to its exceptionally broad substrate selectivity [18].

Human* EPHX1* gene is located in the long arm of chromosome 1q42.1, consisting of 9 exons spanning approximately 35.48 kbps, and it encodes a protein of 455 amino acids [19].* EPHX1* genetic polymorphisms affect the warfarin maintenance dose and may significantly contribute to interindividual differences in the responses to warfarin [6, 20]. A possible mechanism for the influence of* EPHX1* genetic polymorphisms on warfarin maintenance dosage is that genetic variations in the* EPHX1* gene may be conducive to the weakening of oxidized vitamin K to reduced vitamin K and the decrease of epoxide hydrolase enzyme activity, strongly impacting on the generation of active coagulation factors; therefore, it may be correlated to the efficacy and dose of warfarin [13].

Several common single nucleotide polymorphisms (SNPs) in the* EPHX1* gene have been reported previously for the effects of* EPHX1* genetic polymorphisms on the maintenance doses of warfarin; among these polymorphisms, the most frequent functional polymorphisms are rs4653436 A>G and rs2292566 G>A [14, 21, 22]. Recently, a number of studies have shown that these two common SNPs in the* EPHX1 *gene might be major genetic determinants of warfarin dose [6, 23], but the results of other studies have been inconsistent [13, 21]. In view of the conflicting results from previous studies, we performed a meta-analysis of all available data to investigate the influence of* EPHX1* rs2292566 G>A and rs4653436 A>G polymorphisms on warfarin maintenance dosage.

## 2. Materials and Methods

### 2.1. Literature Search and Selection Criteria

A comprehensive search for related studies published before March 2014 was conducted on* PubMed*,* Embase*,* Web of Science*,* Cochrane Library*,* CISCOM*,* CINAHL*,* Google Scholar*,* China BioMedicine* (CBM), and* China National Knowledge Infrastructure *(CNKI) databases. We used a series of keywords and MeSH terms as follows: [“Epoxide Hydrolases” or “EPHX1 protein, human” or “Microsomal Epoxide Hydrolase” or “Styrene Epoxide Hydrolase”] and [“single nucleotide polymorphism” or “SNP” or “polymorphism” or “mutation” or “mutant” or “variation” or “variant”] and [“Warfarin” or “Coumadin” or “Warfarin Potassium” or “Warfarin Sodium”]. There was no language restriction. We also did a manual search of reference lists from potentially relevant articles to identify other potential studies.

The article "Influence of Two Common Polymorphisms in the EPHX1 Gene on Warfarin Maintenance Dosage: A Meta-Analysis" was retracted in 2019. Reasons: errors in the analysis; plagiarism; overlap with other authors' work; false authorship.

The studies which are in accordance with the following criteria were enrolled in the analysis: (1) clinical study focused on the influence of* EPHX1* rs2292566 G>A and rs4653436 A>G polymorphisms on warfarin maintenance dosage, and the warfarin maintenance dose was defined by the international normalized ratio (INR) measurements [24]; (2) all patients should undergo anticoagulation therapy; (3) the data of genotype frequencies and warfarin maintenance dose should be sufficient. Studies were excluded if they do not meet all of these inclusion criteria. If more than one study by the same author using the same case series was published, not only the study with the largest sample size but also the most recent publication was included. Any disagreements were resolved by discussions and subsequent consensus.

### 2.2. Data Extraction and Methodological Assessment

According to the standardized form, data extraction from each included study was done by two authors. We evaluated the methodological quality of each included study based on the Newcastle-Ottawa Scale (NOS) criteria [25]. Briefly, the overall star assessed three main categories on the following: (1) subject selection: 0~4; (2) comparability of subject: 0~2; (3) clinical outcome: 0~3. NOS scores ranged from 0 to 9; and a score ≥ 7 indicates a good quality.

### 2.3. Statistical Analysis

Meta-analysis was performed with the use of the STATA statistical software (Version 12.0, Stata Corporation, College Station, TX, USA). Standardized mean difference (SMD, Cohen's D) and 95% confidence interval (95% CI) were calculated as estimates of relative risk for warfarin maintenance dose under different genetic models. The *Z* test was used to estimate the statistical significance of pooled SMDs. Heterogeneity among studies was estimated by the Cochran's* Q*-statistic and *I* ^2^ tests [26]. If* Q*-test shows a *P* < 0.05 or *I* ^2^ test exhibits > 50% which indicates significant heterogeneity, the random effects model was conducted, or else the fixed-effects model was used [27]. Meanwhile, if there was significant heterogeneity, subgroup analysis was performed to find potential explanatory variables. In order to evaluate the influence of single studies on the overall estimate, a sensitivity analysis was performed. Funnel plots and Egger's linear regression test were applied to investigate publication bias [28].

The article "Influence of Two Common Polymorphisms in the EPHX1 Gene on Warfarin Maintenance Dosage: A Meta-Analysis" was retracted in 2019. Reasons: errors in the analysis; plagiarism; overlap with other authors' work; false authorship.

## 3. Results

### 3.1. Study Selection and Characteristics of Included Studies

Initially, the highly sensitive search strategy identified 34 articles. We reviewed the titles and abstracts of all articles and excluded 15 articles; full texts were also reviewed and 10 articles were further excluded. One study was also excluded due to the lack of data integrity. Finally, 7 cohort studies with a total of 2,063 subjects met our inclusion criteria for qualitative data analysis [6, 13, 14, 20, 21, 23, 29–38].  Figure 1 shows the selection process of eligible articles. Publication years of the eligible studies ranged from 2010 to 2013. Distribution of the number of topic-related literatures in the electronic database during the last decade is shown in Figure 2. Overall, 3 studies were conducted among Caucasians and 4 studies among Asians. LightSNiP assay, SNaPshot assay, DHPLC, TaqMan assay, and base-quenched probe were used for genotyping. NOS scores of all included studies were ≥5. We summarized the study characteristics and methodological quality in Table 1.

### 3.2. Quantitative Data Synthesis

Meta-analysis results illustrated that* EPHX1* rs2292566 G>A polymorphism might be an underlying factor for increased maintenance doses of warfarin with warfarin maintenance dosage higher in individual with* EPHX1* rs2292566 G>A mutation (GG versus AA: SMD = 0.76, 95% CI: 0.47~1.05, and *P* < 0.001; GG versus GA: SMD = 0.43, 95% CI: 0.03~0.83, and *P* = 0.035, resp.), while a similar result was not detected in the comparison of GA versus AA in the* EPHX1* rs2292566 G>A mutation (SMD = 0.31, 95% CI: −0.15~0.76, and *P* = 0.186). However, no significant interaction of* EPHX1* rs4653436 polymorphism with warfarin maintenance dosage was detected (AA versus GG: SMD = −0.01, 95% CI: −0.33~0.32, and *P* = 0.974; AA versus AG: SMD = 0.10, 95% CI: −0.05~0.24, and *P* = 0.209; and AG versus GG: SMD = −0.21, 95% CI: −0.46~0.03, and *P* = 0.092, resp.) (Figure 3).

We also conducted subgroup analyses to investigate the influence of potential factors on individual variability in warfarin dose. As shown in Figure 4, the final triangle is the weighted outcome across groups. Although no significant heterogeneity was found in most parts of those ethnic subgroups, we still continue our subgroup analysis for a secondary verification of our results. Five in all enrolled studies supplied the results of subgroup analysis based on ethnicity, indicating that* EPHX1* rs2292566 G>A polymorphism was associated with warfarin maintenance dosage among Caucasians (GG versus AA: SMD = 0.52, 95% CI: 0.07~1.03, and *P* = 0.006; GG versus GA: SMD = 0.28, 95% CI: 0.07~0.49, and *P* = 0.009, resp.), but not Asians (all *P* > 0.05) (Figure 4). Nevertheless, we observed no associations between* EPHX1* rs4653436 A>G polymorphism and warfarin maintenance dosage among both Caucasians and Asians (all *P* > 0.05). Further subgroup analyses based on sample size and genotyping method revealed significant relationships between* EPHX1* rs2292566 G>A polymorphism and an increased warfarin maintenance dosage in the large-sample-size and TaqMan assay subgroups, but not in the small-sample-size and non-TaqMan assay subgroups (as shown in Table 2). Nevertheless, we also observed no correlations between* EPHX1* rs4653436 A>G polymorphism and warfarin maintenance dosage in all these subgroups (all *P* > 0.05). Sensitivity analysis suggested that no single study could influence the pooled SMDs. Funnel plots demonstrated no evidence of obvious asymmetry existing. The Egger test also did not display strong statistical evidence for publication bias (all *P* > 0.05) (Figure 5).

The article "Influence of Two Common Polymorphisms in the EPHX1 Gene on Warfarin Maintenance Dosage: A Meta-Analysis" was retracted in 2019. Reasons: errors in the analysis; plagiarism; overlap with other authors' work; false authorship.

## 4. Discussion

EPHX1 is putative subunit of the vitamin K epoxide reductase (VKOR) and suggested to be a new genetic variant affecting the warfarin maintenance dose significantly [14, 20]. Generally, through interference with the recycling of vitamin K in the liver, warfarin acts and leads to the secretion of inactive vitamin K-dependent proteins [39]. Warfarin and this vitamin K clotting factors participated in the process of biotransformation formed warfarin interactive pathways [40]. In such progression, vitamin K hydroquinone is oxidized to vitamin K epoxide which is recycled by VKOR to vitamin K and in turn is reduced to vitamin K hydroquinone stimulated by VKOR complex and epoxide hydrolase [41]. Within the vitamin K redox cycle, warfarin suppresses the action of VKOR enzyme complex, partially blocking cycle activity, resulting in the accumulated inactive hepatic vitamin K_1_ 2,3-epoxide and reduced vitamin K depletion [42]. Since this form of vitamin K is an essential cofactor for *γ*-carboxylation of vitamin K-dependent clotting factors, its depletion may lead to a reduction of the active clotting factors [43]. As a matter of fact, a changed dosage intake of the fat-soluble vitamin K can reverse the action of warfarin [44]. Therefore, EPHX1 can be regarded as the other components of VKOR complex involved in the redox processes, so* EPHX1* genetic variations may be crucial candidates in the influence of warfarin anticoagulant effect [45].

The article "Influence of Two Common Polymorphisms in the EPHX1 Gene on Warfarin Maintenance Dosage: A Meta-Analysis" was retracted in 2019. Reasons: errors in the analysis; plagiarism; overlap with other authors' work; false authorship.

In the present meta-analysis, we investigated the relationship between two common SNPs (rs2292566 G>A and rs4653436 A>G) in the* EPHX1* gene and the warfarin dose requirement. Our findings showed a strong association between* EPHX1* rs2292566 G>A polymorphism and warfarin maintenance dose, but similar association was not observed in the* EPHX1* rs4653436 A>G polymorphism, implicating that* EPHX1* rs2292566 polymorphism may be a significant predictor for the interindividual variability of warfarin maintenance dose. Nevertheless, the precise mechanisms that* EPHX1* genetic polymorphisms affect the requirement of warfarin dose are still unidentified. One possible explanation could be that genetic mutations in the* EPHX1 *gene may result in amino acid substitution and have some impacts on the EPHX1 enzyme activity, with resultant impaired warfarin metabolism and clearance, thus contributing to interindividual dose variability [13, 46]. Pautas et al. have identified* EPHX1* rs2292566 G>A polymorphism as a novel predicting factor for variable warfarin response, reporting that alteration in the* EPHX1* gene may change the pharmacokinetics and pharmacodynamics of warfarin exertion by inhibiting the activity of vitamin K epoxide reductase (VKOR), and thereby may influence warfarin maintenance dose [14]. Loebstein et al. have revealed that VKOR was involved in vitamin K redox cycle, and VKOR plays a crucial role in promoting inactive vitamin K into active vitamin K, which is an essential cofactor for *γ*-carboxylation of vitamin K-dependent clotting factors in the hepatic system (II, VII, IX, and X) [42]. Furthermore, a previous study identified* EPHX1* genetic variant as a predictor of variable warfarin dose requirement because* EPHX1* has been proposed as a putative subunit of VKOR [44]. Therefore, it seems reasonable to hypothesize that* EPHX1* rs2292566 G>A polymorphism may reduce VKOR activity and consequently give rise to active vitamin K deficiency, which may lead to a decrease of the active clotting factors. Additionally, it is plausible that patients with* EPHX1* rs2292566 polymorphism may require a lower maintenance dose of warfarin. Furthermore, it should be noted that out of those six forest plots, there were only significant relationships between the comparison of GG versus AA and GG versus GA; no potential association was detected from the GA versus AA comparison in the* EPHX1* rs2292566 G>A polymorphism; one possible explanation is that the existence of possible heterogeneity sources could have an influence on the overall outcome, so no significant relationship was observed between dose variations and certain allele types for the differences in ages or ethnic backgrounds [20]. Our results are in line with a recent cohort study, which genotyped 107 patients who had stable doses and INRs at their last three consecutive visits and displayed that* EPHX1* rs2292566 G>A polymorphism was significantly associated with the warfarin maintenance dose, accounting for 1.7% of the variability in the dose [20].

The article "Influence of Two Common Polymorphisms in the EPHX1 Gene on Warfarin Maintenance Dosage: A Meta-Analysis" was retracted in 2019. Reasons: errors in the analysis; plagiarism; overlap with other authors' work; false authorship.

Considering the possibility of existing obvious heterogeneity, which may negatively affect our association study results, stratified analyses were carefully performed based on ethnicity, genotyping method, and sample size. Subgroup analysis after the heterogeneity test was also a required step for the secondary verification of our results. The results of subgroup analysis performed by ethnicity displayed significant associations between* EPHX1* rs2292566 G>A polymorphism and a lower maintenance dose of warfarin in Caucasians, while no similar association was detected among Asians, implicating that ethnicity differences may play an important role in the effects of variants in the* EPHX1* gene on interindividual variability of warfarin maintenance dose. Although the potential mechanism of ethnicity differences is still not fully understood, we supposed that ethnicity may result in differences in alleles and genotypes among different ethnic populations. Sample size within those included papers were obviously different, and this stratified analysis revealed that a significant difference between* EPHX1* rs2292566 G>A polymorphism and warfarin maintenance dose was observed within the larger sample sizes. In summary, our findings are consistent with the previous studies that* EPHX1* rs2292566 G>A polymorphism may influence the warfarin dose requirement, suggesting that translation of this knowledge into clinical guidelines may offer a useful and informative route to improve therapeutic management during warfarin therapy.

The current meta-analysis also had several limitations that should be acknowledged. First, our results lacked sufficient statistical power to assess the correlations of* EPHX1* genetic polymorphisms with the warfarin dose requirements. Secondly, meta-analysis is a retrospective study that may inevitably induce subject selection bias and thereby have an impact on the reliability of our results. Thirdly, our meta-analysis failed to obtain original data from the included studies, which may limit further evaluation of potential role of* EPHX1* genetic polymorphisms with the warfarin dose requirements.

The article "Influence of Two Common Polymorphisms in the EPHX1 Gene on Warfarin Maintenance Dosage: A Meta-Analysis" was retracted in 2019. Reasons: errors in the analysis; plagiarism; overlap with other authors' work; false authorship.

In conclusion, our meta-analysis provides robust and unambiguous evidence that* EPHX1* rs2292566 G>A polymorphism may affect the maintenance dose of warfarin in Caucasians, so* EPHX1* rs2292566 G>A polymorphism could be a potential and practical biomarker for the interindividual variability of warfarin maintenance dose. However, due to the limitations mentioned above, more reliable research with larger sample sizes is still required to provide a more comprehensive and representative statistical analysis precisely.

## Figures and Tables

**Figure 1:** Flow chart shows study selection procedure. Seven cohort studies were included in this meta-analysis.

**Figure 2:** The distribution of the number of topic-related literatures in the electronic database during the last decade.

**Figure 3:** Forest plots for the relationships of* EPHX1* rs2292566 G>A and rs4653436 A>G polymorphisms with warfarin maintenance dosage. The final triangle is the weighted outcome across groups.

**Figure 4:** Subgroup analyses for the relationships between* EPHX1* rs2292566 G>A polymorphism and warfarin maintenance dosage. The final triangle is the weighted outcome across groups.

**Figure 5:** Funnel plot of publication biases for the relationships between* EPHX1* rs2292566 G>A polymorphism and warfarin maintenance dosage. The final triangle is the weighted outcome across groups.

**Table 1:** Baseline characteristics and methodological quality of all included studies.

First author	Year	Country	Ethnicity	Case number	Gender (M/F)	Age (years)	Genotyping method	SNP	NOS score
Özer [20]	2013	Turkey	Asians	107	53/54	53.9 ± 13.6	LightSNiP assay	rs2292566 G>A	6
Liang [6]	2013	China	Asians	300	138/162	47.9 ± 12.5	SNaPshot assay	rs2292566 G>A	8
								rs4653436 A>G	8
Volcik [37]	2006	China	Asians	217	90/127	51.3 ± 15.0	DHPLC	rs4653436 A>G	7
Ciccacci [21]	2011	Italy	Caucasians	141	78/70	68.2	TaqMan	rs2292566 G>A	6
								rs4653436 A>G	6
Luo [23]	2010	China	Asians	197	82/115	52.9 ± 11.8	Base-quenched probe	rs2292566 G>A	7
								rs4653436 A>G	7
Pautas [14]	2010	France	Caucasians	290	69/231	86.7 ± 6.0	TaqMan	rs2292566 G>A	8
Carlquist [13]	2010	USA	Caucasians	168	79/89	71.0 ± 13.0	TaqMan	rs4653436 A>G	7

M: male; F: female; DHPLC: denaturing high performance liquid chromatography; NOS: Newcastle-Ottawa Scale criteria; SNP: single nucleotide polymorphisms.

**Table 2:** Meta-analysis of the associations between *EPHX1* rs2292566 G>A polymorphism and warfarin maintenance dosage.

	GG versus AA					GG versus GA					GA versus AA				
	SMD	95% CI	*P*	*P*_*h*_	*I* ^2^	SMD	95% CI	*P*	*P*_*h*_	*I* ^2^	SMD	95% CI	*P*	*P*_*h*_	*I* ^2^
Overall	0.76	0.47~1.05	<0.001	0.699	0.0%	0.43	0.03~0.83	0.035	<0.001	87.6%	0.31	−0.15~0.76	0.186	0.105	47.7%
Ethnicity															
Caucasians	0.52	0.07~1.03	0.006	0.716	0.0%	0.28	0.07~0.49	0.009	0.550	0.0%	0.40	−0.25~1.06	0.226	0.028	72.0%
Asians	0.84	−0.13~1.15	0.699	0.895	0.0%	0.54	−0.14~1.23	0.122	<0.001	92.6%	0.05	−0.72~0.82	0.898	0.830	0.0%
Sample size															
Small (*n* < 300)	0.71	−0.01~1.10	0.310	0.462	0.0%	0.24	−0.13~0.60	0.210	0.058	64.8%	−0.05	−0.46~0.36	0.815	0.724	0.0%
Large (*n* ≥ 300)	0.82	0.40~1.24	<0.001	0.479	0.0%	0.67	0.01~1.34	0.042	<0.001	93.0%	0.62	0.17~1.07	0.007	0.334	8.7%
Genotyping method															
TaqMan assay	0.78	0.02~1.03	0.465	0.716	0.0%	0.28	0.07~0.49	0.009	0.550	92.6%	0.40	−0.25~1.06	0.226	0.028	72.0%
Non-TaqMan assay	0.84	0.00~1.15	0.051	0.895	0.0%	0.54	−0.14~1.23	0.122	<0.001	0.0%	0.05	−0.72~0.82	0.898	0.830	0.0%

*EPHX1*: epoxide hydrolase 1; SMD: standardized mean difference; 95% CI: 95% confidence interval; *P*_*h*_: the *P* value for the heterogeneity test.
